The article "Treatment Effect of Type 2 Diabetes Patients in Outpatient Department Based on Blockchain Electronic Mobile Medical App" was retracted in 2023. Reasons: unreliable results or conclusions; lack of ethics approval or compliance; concerns about the data; concerns about the peer review.

# Treatment Effect of Type 2 Diabetes Patients in Outpatient Department Based on Blockchain Electronic Mobile Medical App

**DOI:** 10.1155/2021/6693810

**Published:** 2021-03-01

**Authors:** Yang Liu, Zhaoxiang Yu, Hua Sun

**Affiliations:** ^1^Department of Endocrine, Affiliated Hospital of Beihua University, Jilin 132012, China; ^2^Department of Anesthesiology, Affiliated Hospital of Beihua University, Jilin 132012, China

## Abstract

As the pace of people's lives accelerates, there are more and more diabetic patients. This research mainly explores the treatment effect of type 2 diabetic patients based on blockchain electronic mobile medical app. Considering that it is more realistic to adopt an off-chain storage solution, the blockchain-based medical data sharing platform in this study adopts an off-chain storage solution. Only key information is stored in the blockchain network, and all medical data will be in the cloud space. For storage, cloud storage uses Aliyun's OSS storage service, which can be expanded infinitely. The cloud operation module is responsible for all operations that interact with cloud storage. The chain code can call the cloud operation module to upload the user's encrypted medical data and user ID to Alibaba Cloud's OSS. The chain code will return the storage address of the medical data and the authorized access address is sent to the blockchain network for consensus on the chain. The message processing module provides information processing functions such as chat information processing, APP use reminders, and health tips. The indicator recording module includes indicator recording functions including 6 indicators of blood sugar, medication, diet, weight, exercise, and sleep. The main function of the indicator analysis module is to display the curve trends of the 6 indicators recorded by the patient in three days, one week, and one month. Comparing the change range of the mean value of glycosylated hemoglobin at the beginning and end of the two groups of patients, it can be found that the change range of glycosylated hemoglobin in the intervention group is −6.04%, while the change range of the control group is only −3.26%. The impact of the mobile medical app designed in this study will indeed be reflected in the patient's blood sugar control and help patients to better control blood sugar.

## 1. Introduction

China's public health and medical institutions sounded the alarm [1]. Diabetes is an incurable but controllable chronic lifelong disease. The treatment of diabetes should not only stop at short-term diagnosis and treatment control standards. Long-term, stable, and safe hypoglycemic plan is the goal we should pursue, which will help. In order to delay the occurrence and development of chronic complications of diabetes, the emergence of mobile phone APP has made the long-term chronic health management of type 2 diabetes traceable, which is bound to promote the development of China's public health cause.

The application of medical mobile phone app and doctors' online diagnosis and treatment can help patients control blood sugar within a relatively standard [2], stable, and safe range, and long-term education and guidance facilitate patients to form correct living habits, and the online communication function provides timely communication between doctors and patients and provides a good platform. Long-term high blood sugar has caused a huge spiritual and economic burden on patients, their families, and society. The health management of type 2 diabetes is urgent and has great social significance.

Oxidative stress is considered to be the main mediator of the progression of diabetes complications. Panigrahy believes that intracellular reactive oxygen species (ROS) cause oxidative stress. The reactive oxygen species he increased through these pathways caused *β*-cell dysfunction and insulin resistance, responsible for cell damage and death. Although he proposed a speculative mechanism based on the development of diabetes, he did not summarize ROS as a potential therapeutic target [3]. Mann found that liraglutide can reduce the primary endpoint risk and death. He reported on the predetermined secondary renal outcome of the randomized controlled trial, and the study designated patients to receive liraglutide or placebo. He used intention-to-treat methods to analyze the time of events to determine the risk of renal prognosis. Although he analyzed the changes in the estimated glomerular filtration rate and proteinuria, he did not give specific research data [4]. Xue conducted a cohort study of 24,996 Chinese adults aged 35–74, and 19.9% of the subjects were lost to follow-up. He collected information about diabetes events during his follow-up. He used the population attributable risk adjusted for confounding factors, the incidence of diabetes, and the size of the population in China to estimate the number of T2D events caused by abdominal obesity. The definition of abdominal obesity he proposed has no basis and lacks scientific logic [5]. Eun believes that the severity of nonalcoholic fatty liver disease (NAFLD) in type 2 diabetes (T2DM) has not been assessed. He used the controlled attenuation parameter (CAP) to investigate the prevalence and severity of NAFLD in the T2DM population. He chose the CAP values of 250 dB/m and 300 dB/m as the critical values for the presence of NAFLD and moderate-to-severe NAFLD, respectively. The subjects he included lacked specific standards, and the research process was too complicated [6].

Considering that it is more realistic to adopt an off-chain storage solution, the blockchain-based medical data sharing platform in this study adopts an off-chain storage solution. Only key information is stored in the blockchain network, and all medical data will be in the cloud space. For storage, cloud storage uses Aliyun's OSS storage service, which can be expanded infinitely. The cloud operation module is responsible for all operations that interact with cloud storage. The chain code can call the cloud operation module to upload the user's encrypted medical data and user ID to Alibaba Cloud's OSS. The chain code will return the storage address of the medical data and the authorized access address is sent to the blockchain network for consensus on the chain [7]. The message processing module provides information processing functions such as chat information processing, APP use reminders, and health tips.

## 2. Outpatient Treatment of Type 2 Diabetes

### 2.1. Blockchain Technology

The blockchain uses a timestamp-based chain block structure at the bottom layer to provide nodes in the blockchain network with nonrepudiation results, proving the existence or absence of certain data or state transitions in the blockchain database [8, 9]. As long as the underlying cryptographic primitives (hash functions and signature schemes) are computationally secure or most blockchain maintainers conduct collusion activities, these lines of evidence cannot be forged by third parties through calculations [10]. In addition, the cost for anyone to forge such evidence will be prohibitive, and the forgery itself has long-term undeniability [11, 12].

The consensus mechanism is to ensure that even if the nodes keep separate accounts, they can ensure that the accounts kept by each node will not conflict or contradict [13, 14]. The consensus algorithm is used in the blockchain system to ensure that the database copy that has not been tampered with is the same as the correct database state [15, 16]. That is, the consensus algorithm is used to ensure that the transaction in the log is eventually propagated to all normal operating nodes in the blockchain network and to ensure that the changes produced on all normal operating nodes are consistent [17]. The consensus algorithm can be used not only as a means of identification but also as a means to prevent tampering [18, 19]. The consensus algorithm is one of the core parts of the blockchain, and different consensus algorithms have different security and efficiency [20]. Blockchain can deploy different company algorithms according to different usage scenarios with different efficiency and security requirements to ensure a good user experience [21, 22]. The basic model of the blockchain is shown in Figure 1.

Assuming that the existing *k* voting nodes have signed (that is, voted) the message of a certain production node, we have that

(1) Rsourse=⊕i=0k−1Signaturei⊕Timestramp,Q=StrToIntSubStrEnd32HmodMQ,

where *Q* is a random number [23]. Assuming that it casts *K* votes in each round of recurring calculations and casts them to *K* nodes, then each node is voted with the probability of PI:

(2) $$\begin{array}{c} P1=\frac{K}{\text{Md}}\text{.} \end{array}$$

Then, assuming that each node gets *Y* votes with probability *P*2, we can get

(3) $$\begin{array}{c} P2=C_{MW}^{Y}*\left(\frac{K}{\text{Md}}\right)*{\left(1-\frac{K}{\text{Md}}\right)}^{\text{Md}-Y}. \end{array}$$

Assuming that the probability of being successfully selected as a production node is *P*3, we get

(4) $$\begin{array}{c} P3=\overset{Mw}{\underset{i=Mw/2}{\sum }}\frac{Mw!}{\left(i!\left(Mw-i\right)!\right)}*{\left(\frac{K}{\text{Md}}\right)}^{i}*{\left(1-\frac{K}{\text{Md}}\right)}^{Mw-i}. \end{array}$$

The system selects Mq production nodes from Md candidate nodes. Then, let *P*4 be the probability that the candidate node is successfully selected as a production node; namely,

(5) $$\begin{array}{c} P4=\frac{\text{Mq}}{\text{Md}}. \end{array}$$

When *P*3=*P*4, *K* can be calculated [24, 25].

### 2.2. App User Experience Evaluation Indicators

It needs to be nondimensionalized, that is, by dividing the k column to adjust the sequence to ensure that the evaluation scores of all the sequence are in the interval (0, 1) [26].

(6) $$\begin{array}{c} f\left(X_{i}\left(k\right)\right)=\frac{X_{i}\left(k\right)}{A\left(k\right)},\\ X_{i}=\left(X_{1i},X_{2i},\ldots ,X_{ji}\right),\;i=1,2,\ldots ,n. \end{array}$$

According to the results of the questionnaire evaluation, a judgment matrix of *n* evaluation indicators can be obtained, among which *C*1, *C*2, *C*3 … *C*n are the evaluation indicators of the medical app user experience [27, 28].

(7) $$\begin{array}{c} A={\left(a_{ij}\right)}_{m\times n}=\begin{array}{c} C1\\ C2\\ \vdots \\ Cn \end{array}\left[\begin{array}{cccc} a_{11} & a_{12} & \cdots & a_{1n}\\ a_{21} & a_{22} & \cdots & a_{2n}\\ \vdots & \vdots & \vdots & \vdots \\ a_{n1} & a_{n2} & \cdots & a_{nn} \end{array}\right]. \end{array}$$

The importance of the project *C*_i_ relative to *C*_j_ can be expressed as

(8) $$\begin{array}{c} a_{ij}=\frac{w_{i}}{w_{j}}. \end{array}$$

Its determinant can be expressed as

(9) $$\begin{array}{c} A=\left[\begin{array}{ccc} \frac{w_{1}}{w_{1}} & \cdots & \frac{w_{1}}{w_{n}}\\ \vdots & \vdots & \vdots \\ \frac{w_{n}}{w_{1}} & \cdots & \frac{w_{n}}{w_{n}} \end{array}\right],\\ W=\left[\begin{array}{c} w_{1}\\ \cdots \\ w_{n} \end{array}\right]. \end{array}$$

Therefore,

(10) $$\begin{array}{c} w_{i}=\frac{1}{n}\sum_{j=1}^{n}\frac{a_{ij}}{\sum_{i=1}^{n}a_{ij}},\;i,j=1,2,3\ldots n. \end{array}$$

*W* in the matrix is the eigenvector of *A* [27]. Due to minor changes, we have

(11) $$\begin{array}{c} \text{CI}=\frac{\lambda_{\max}-n}{n-1}. \end{array}$$

The smaller the CI value, the higher the consistency. The consistency of randomly generated upside-down matrices is called  RI. When the order is the same, the ratio of CI to RI is called the consistency ratio CR:

(12) $$\begin{array}{c} \text{CR}=\frac{\text{CI}}{\text{RI}}. \end{array}$$

All the weight results that pass the consistency test are grouped to obtain the final weight coefficient w_*i*_^*G*^ for each indicator [29].

(13) $$\begin{array}{c} w_{i}^{G}={\prod_{k=1}^{K}\left[w_{i}^{k}\right]}^{a_{k}},\;i=1,2,\ldots ,n. \end{array}$$

## 3. Outpatient Treatment Experiment of Type 2 Diabetes

### 3.1. Smart Contract Design and Implementation

#### 3.1.1. Adding Medical Data

When the system calls the chain code to add medical data, adding a medical data contract will first collect the medical data information filled in by the user from the WEB backend and then use the medical data information filled in by the user to perform medical data through the medical data value prediction model in the public service module value prediction; after receiving the predicted value given by the medical data value prediction model [30], the data value is added to the medical data information and the user's complete medical data is encrypted through the encryption service in the public service module, and then the public service module is called. The cloud storage service in China uploads the complete encrypted data to the cloud and at the same time obtains the storage address and authorized access link of the data in the cloud, adds it to the key information of the medical data, and finally sends all the key information of the medical data to the blockchain consensus on the chain in the network.

#### 3.1.2. Medical Data Update

When the system calls the chain code to update the medical data, the chain code will first request relevant data key information from the blockchain network. After the relevant data key information is queried by the blockchain, it will return the corresponding data key information to the chain code. The code can then download the corresponding encrypted data through the cloud storage module in the public service module according to the returned key information of the relevant data. After the encrypted medical data are successfully downloaded, the chain code will call the decryption service in the public service module to perform the downloaded medical data. Decrypt and display it to the user through the WEB backend for viewing, and wait for the user to make corresponding updates to the medical data information [31]. After the user completes the update of the medical data, the chain code will read the user's basic medical information again from the WEB backend. Call the medical data value prediction model in the public service module to predict the value of the data. After receiving the data value given by the medical data value prediction model, the complete medical data are encrypted through the encryption service in the public service module. Through the cloud storage service in the public service module, the complete encrypted medical data are stored in the cloud. After receiving the medical data cloud storage address and the medical data authorized access link returned by the cloud storage service, all key data information is sent to the district. The blockchain network performs consensus on the chain and completes the update of data.

#### 3.1.3. Viewing Medical Data

When the system calls to view all medical data chain codes, the chain code will first request the blockchain network to view all key medical data information. After receiving all the key medical data information obtained by the blockchain network, the chain code can be based on the key information of medical data returned by the blockchain network which is downloaded through the cloud storage service in the public service module. After the complete medical data encryption service is successfully downloaded, the chain code can call the medical data decryption service in the public service module. Decrypt the data. After the decryption is successful, the medical data can be sent to the WEB backend for users to view. When the data purchaser is used to view all legal and valid medical data information that has been uploaded to the platform, the WEB backend will be based on the medical data. The legality of the information is screened. The data purchaser cannot see the medical data that is temporarily illegal and invalid. The data auditor can view all medical data, whether legal or illegal, and can call them according to the actual situation of the medical data. The verification medical data chain code is used to mark the validity of the data.

#### 3.1.4. Personal Medical Data Call

When the system calls to view the personal medical data chain code, the chain code will first send the key information of the individual user to the blockchain network. The blockchain network will query the key information of the relevant medical data based on the key information of the individual user sent by the chain code. The relevant information is returned to the chain code, and then the chain code can download personal encrypted medical data through the cloud storage service in the public service module according to the data storage address in the medical data key returned by the blockchain network. After the medical data, the chain code can call the decryption service in the public service module to decrypt the encrypted personal medical data. After successful decryption, the chain code will send the decrypted personal medical data to the WEB backend for users to view the medical data information for the next step.

#### 3.1.5. Call Authorized Medical Data

When the system calls the authorized medical data chain code, the chain code will request the key information of the personal medical data from the blockchain network. After receiving the key information of the medical data queried by the blockchain network based on the personal information, the chain code will call the public service cloud storage module and the module downloads the encrypted personal medical data according to the medical data storage address in the medical data key information returned by the blockchain network. After successfully downloading the encrypted medical data, the chain code will call the decryption service in the public service module. Decrypt the downloaded encrypted personal medical data. After the decryption is successful, the chain code will send the decrypted medical data to the WEB backend for users to view. The user can authorize the personal medical data or not after viewing the personal medical data. Authorize instructions and send the corresponding instructions together with the key information of personal medical data to the blockchain network for consensus on the chain operation [32].

### 3.2. Design and Implementation of Cloud Operation Module

Because the nodes in the blockchain network do not store the user's complete data information but only store the metadata, if the system is attacked, only the metadata may be completely preserved, and the data itself will be completely lost. Considering that it is more realistic to adopt an off-chain storage solution, the blockchain-based medical data sharing platform in this article also uses an off-chain storage solution. Only key information is stored in the blockchain network, and all medical data will be in the cloud space. For storage, cloud storage uses Aliyun's OSS storage service, which can be expanded infinitely. OSS is more in line with the actual application scenarios of the data sharing platform in this article. Therefore, all medical data in this platform's off-chain storage solution will be stored using Alibaba Cloud's OSS standard storage services. The cloud operation module is responsible for all operations that interact with cloud storage. The chain code can call the cloud operation module to upload the user's encrypted medical data and the user's ID to Alibaba Cloud's OSS [33] and return the storage address and authorized access address of the medical data to the chain code after successful storage, and the chain code will return. The storage address and authorized access address of the medical data are sent to the blockchain network for consensus uploading.

### 3.3. Mobile Medical App Function Design

1. Message processing module: this module provides information processing functions such as chat information processing, APP use reminders, and health tips. Among them, chat information includes three types of patient group chat information, individual chat information between patients, and chat information between patients and doctors. App reminders include information to remind patients to use various index recording functions and chat functions. Health tips are a regular update of health knowledge on Mondays, Wednesdays, and Fridays.
2. Indicator recording module: this module includes index recording functions including 6 indexes of blood sugar, medication, diet, weight, exercise, and sleep. Among them, for blood glucose records, patients can choose 8 time periods, including early morning, before breakfast, and after breakfast. In exercise recording, patients can choose five types of activities such as walking/fast running, square dancing/gymnastics to record exercise time, and exercise time, respectively [34]. In the diet record, it is also possible to record the consumption of foods such as cereals and fruits in the breakfast, lunch, and dinner or upload photos to be identified by the computer. Medication records and weight records are regardless of time period. In addition, since patients may forget to record, the module also supports patients to make up-entry of records in the past period of time.
3. Indicator analysis module: the main function of this module is to display the curve trend of the 6 indicators recorded by the patient in three days, one week, and one month. Among them, blood glucose analysis can choose the early morning, before breakfast, and other time periods to analyze the graph. Weight analysis can calculate the corresponding body mass index (BMI) value based on the patient's weight and height. In the diet analysis, the curve changes of the food intake in the minutes of breakfast, lunch, and dinner can be displayed, respectively. At the same time, in the analysis of these six indicators, when the patient's data is higher or lower than the highest or lowest value of the normal health range, an upward or downward arrow will be displayed to remind the patient to pay attention. In addition, patients can see the indicator analysis curves of other patients in the same group, understand the health management of other patients, and play a certain incentive role.

### 3.4. Intervention Plan Design

Before the trial, all patients were given diabetes-related education, including healthy eating methods, healthy exercise methods, effective blood glucose monitoring methods and procedures, oral medication misunderstandings, precautions for insulin preservation and injection, and complications prevention methods. The patients were handed out health handbooks and small gifts. The patients who clearly expressed interest in the project were instructed to fill in the baseline questionnaire and perform the baseline glycosylated hemoglobin test. In addition, for patients in the intervention group, the researchers will download the APP and train them to ensure that they will use all the functions of the APP, such as recording blood sugar, viewing health knowledge, and online communication and open accounts and permissions for them.

During the trial, the hospital doctors provided two groups of patients with offline diabetes knowledge education twice a month. The main forms of education were PPT lectures, doctor-patient interaction, health knowledge questions and answers and so forth to mobilize patients' self-management. In addition to participating in offline health education, patients in the intervention group continued to use APP for online self-management, that is, to record and view various indicators. In addition, patients can also communicate with doctors and patients online, and the content of online consultations for patients will be answered regularly by doctors in a hospital. Patients in the intervention group can also view health knowledge in the APP, including knowledge about diabetes complications, diet, exercise, and so forth. The update frequency of health knowledge is every Monday, Wednesday, and Friday, and health knowledge updates will be sent to patients in the APP to remind them to check their health knowledge.

After the trial, the end-of-term questionnaire survey was conducted again on the two groups of patients, and the second HbA1c test was conducted. At the same time, according to the comprehensive performance of the two groups of patients within 3 months, gifts were given to patients with higher cooperation and better performance. The variables and measurement methods are shown in Table 1.

## 4. Treatment of Type 2 Diabetes Patients in Outpatient Department

### 4.1. Sociodemographic Characteristics before Intervention

According to the analysis of independent-sample *t*-test and chi-square test, the difference in age and gender between the two groups of patients was not significant (*P* > 0.05), and the difference in gender was smaller. At the same time, we found that there are fewer female patients in both groups, which is directly related to the higher proportion of male patients when recruiting patients, and the enthusiasm of male patients and the degree of cooperation with the project are relatively high. In addition to age and gender, it is also necessary to compare the education level, marital status, and position type of the two groups of patients; that is, the chi-square test is used to verify the differences in the proportions of various indicators between the two groups. The results showed that, in terms of educational level, most of the patients in the two groups were at the level of high school/technical school. Relatively speaking, patients in the intervention group had a higher educational level. There were certain differences between the two groups, but the *P* value was close to 0.05; that is, the difference is small. In terms of marital status, due to the age of the two groups of patients, 80%–90% of the patients are married, and the job types are mainly ordinary employees and retired employees, both of which are closely related to the age of the patients. The results showed that the two groups of patients had no significant difference in these two indicators (*P* > 0.05), and they were completely comparable. The age comparison between the two groups of patients before the intervention is shown in Table 2. Other demographic characteristics of the two groups of patients are shown in Table 3. The analysis of other demographic characteristics of patients is shown in Figure 2.

The basic situation of the disease before the intervention is shown in Figure 3. This section will compare the disease conditions of the two groups of patients, including the patient's course of disease, number of complications, medication methods, whether to use other health management software, and how to record their own indicators. Since the course of disease and the number of complications belong to the continuous attribute, the independent-sample *t*-test was used to compare the differences. The comparison results are shown in Table 4. About 89.5% of patients in the intervention group had 0–2 complications, and about 81.1% of the patients in the control group had 0–2 complications. Therefore, the number of complications in the intervention group was slightly higher than that in the control group. Similarly, in the course of illness, patients in the intervention group are also slightly more than those in the control group, which reflects from the side that the longer the course of the patient, the higher the number of complications. The chi-square test was used to verify the differences between the groups. Patients in the intervention group and the control group focused on oral medication and medium- and long-acting insulin. The vast majority of patients do not use other management software, only 2 patients use it, and about 70% of patients do not have the habit of recording their own indicators. In general, there was no significant difference in the performance of the two groups of patients on these three indicators (*P* > 0.05).

### 4.2. Comparison of Indicators between the Two Groups of Patients after Intervention

After 3 months, that is, 12 weeks, we conducted a final questionnaire survey on the two groups of patients and performed HbA1c test again to determine the degree of changes in various indicators of the patients during the 3-month period. This questionnaire survey no longer involves the patient's sociodemographic survey form and the disease status survey form but focuses more on measuring the indicators that will change during the trial period. For patients in the intervention group and the control group, after a period of intervention treatment, that is, regular patient education and mobile medical app intervention, the patients may have certain psychological and behavioral changes. For example, patients will realize that there are certain misunderstandings in their existing self-management methods and will improve in actual actions. The comparison of self-efficacy at the end of the two groups is shown in Table 5. According to the comparison results, we found that the final self-efficacy scores of the two groups of patients have a small increase compared with the initial self-efficacy scores. Among them, the range of change in the intervention group was 4.57%, while that in the control group was 3.13%, which indicates that the intervention program in this study had a positive impact on both groups of patients, but the self-efficacy score of the intervention group changed more. The specific changes are shown in Figure 4. In addition, we found that there was basically no difference in the initial self-efficacy scores of the two groups of patients, while the final self-efficacy scores were significantly different (*P* < 0.05). During the intervention period, the only difference between the two groups of patients was whether to use APP for self-management. Therefore, this result shows that mobile medical app has a positive and significant impact on the self-efficacy of patients in the intervention group, which can make patients more confident that they can achieve effective self-management.

### 4.3. Self-Efficacy Changes between the Two Groups

We compared the end-of-term self-management behaviors of the two groups of patients, that is, compared their total scores and the changes in the scores of each subitem and explored whether the mobile medical app has a significant impact on the patients' offline self-management behavior self-evaluation scores to confirm whether the mobile medical app has a significant impact on the patient's daily self-management behavior. The comparison of the change range is shown in Figure 5. It can be found that the mean self-management score of the control group has decreased compared with the beginning of the period, while the intervention group has shown an increase. Among them, the range of change in the intervention group was 0.98%, and the range of change in the control group was −146%. This change was more obvious than the change in self-efficacy. Similarly, in the end-of-term self-management behavior scores of the two groups of patients, we can also find that there is no significant difference at the beginning of the period to a significant difference. This shows that patients' self-management behavior is also positively affected by mobile medical app; that is, the use of mobile medical app makes patients pay more attention to their self-management, and this change is also reflected in their actual actions.

In addition, we want to confirm the main changes in the patient's self-management behavior. Therefore, this article further compares the final scores of each subitem in the self-management behavior of the two groups of patients. The specific comparison is shown in Table 6. From Table 6, we can find that the end-of-term comprehensive management scores of the two groups of patients (that is, the combination of healthy diet, compliance with medical drugs, and exercise) are significantly different. However, there is no obvious difference in these three subitems, which may be caused by the inconspicuous changes in the scores of each subitem. Relatively speaking, the scores of the two groups of patients at the end of the light exercise changed significantly, from 0.7 and 0.78 to 0.82 and 0.81, respectively, which shows that the patients focused on strengthening their own light aerobic exercise. The end-of-term compliance scores of patients in the intervention group also improved. In addition, we found that the end-of-period blood glucose monitoring of the two groups of patients has a more significant difference compared with the beginning of the period (*P* value changed from 0.054 to 0.021), but this difference is mainly manifested in the decrease in the average score of the control group, while in the intervention group there is little change. Based on the above situation, we can find that the influence of mobile medical app on patients' self-management behavior is mainly reflected in the improvement of their exercise and blood glucose monitoring frequency. The patient's self-management analysis is shown in Figure 6.

### 4.4. Blood Glucose Control after Intervention

The changes in patients' self-efficacy and self-management behaviors will largely affect the patient's blood sugar control. Therefore, this section compares the HbA1c values of the two groups of patients after the intervention and compares them with the baseline data of the two groups of patients at the beginning of the period. The results are shown in Table 7. We found that although the HbA1c of the two groups of patients decreased at the end of the period, the difference between the two groups was still not significant after the intervention. This shows that, for patients with diabetes, diabetes education helps patients understand more health knowledge and adjust their own behavior in time to achieve better blood sugar control. The application of mobile medical app will also improve the patient's blood sugar control, but there is no significant difference in the glycosylated hemoglobin of the two groups of patients.

In order to further confirm the effect of mobile medical app on the blood sugar control effect of patients, we compared the change range of the mean value of glycosylated hemoglobin at the beginning and end of the two groups of patients. The comparison results are shown in Figure 7. We can find that the change range of glycosylated hemoglobin in the intervention group is −6.04%, while the change range in the control group is only −3.26%. This shows that the impact of mobile medical app will indeed be reflected in the patient's blood sugar control, and, to a certain positive effect, it will help patients to control blood sugar better.

## 5. Conclusion

When the system calls the chain code to add medical data, adding a medical data contract will first collect the medical data information filled in by the user from the WEB backend and then use the medical data information filled in by the user to perform medical data through the medical data value prediction model in the public service module value prediction; after receiving the predicted value given by the medical data value prediction model, the data value is added to the medical data information and the user's complete medical data is encrypted through the encryption service in the public service module, and then the public service module is called. The cloud storage service in uploading completes encrypted data to the cloud.

When the system calls the chain code to update the medical data, the chain code will first request key information on relevant data from the blockchain network. After the key information on relevant data is queried by the blockchain, it will return the key information on the corresponding data to the chain code. The code can then download the corresponding encrypted data through the cloud storage module in the public service module according to the returned key information of the relevant data. After the encrypted medical data is successfully downloaded, the chain code will call the decryption service in the public service module to perform the downloaded medical data. Decrypt and display it to the user for viewing through the WEB backend, and wait for the user to update the medical data information accordingly.

When the system calls to view all medical data chain codes, the chain code will first request the blockchain network to view all key medical data information. After receiving all the key medical data information obtained by the blockchain network, the chain code can be based on key information of medical data returned by the blockchain network which is downloaded through the cloud storage service in the public service module. After the complete medical data encryption service is successfully downloaded, the chain code can call the medical data decryption service in the public service module. After the decryption is successful, the medical data can be sent to the WEB backend for users to view.

## Figures and Tables

**Figure 1:** Basic model of blockchain.

**Figure 2:** Analysis of other demographic characteristics of patients.

**Figure 3:** Comparison of basic conditions of diseases before intervention.

**Figure 4:** Changes in self-efficacy scores of patients in the intervention group.

**Figure 5:** Comparison of the magnitude of change.

**Figure 6:** Patient self-management.

**Figure 7:** Research comparison results.

**Table 1:** Variables and measurement methods.

Variable name	Variable meaning	Measuring tools	Measure
Old	Age	Survey of sociodemographic characteristics of diabetic patients	Patient age
Gender	Gender		Patient gender (1: male; 2: female)
Education	Education level		Patient education level (1: above elementary school)
Marriage	Marital status		Patient's marital status (1: unmarried; 2: married)
Position	Position		Patient's current position (1: general employee; 2: cadre)
Illness years	Course of illness		As of 2019, the number of years the patient has been sick

**Table 2:** Comparison of the age of the two groups of patients before the intervention.

Variable name	Variable meaning	Intervention group (*N* = 37)	Control group (*N* = 38)	*T*	*P*
Old	Age	56.57 ± 8.73	60.03 ± 7.79	−1.812	0.074

**Table 3:** Comparison of other demographic characteristics of the two groups of patients.

Variable name	Variable	Intervention group (*N* = 37)	Control group (*N* = 38)	*P*
		*N*	(%)	
Gender	1 (male)	12	67.6	0.688
	2 (female)	3	32.4	

Education	1 (primary school and below)	6	8.1	0.043
	2 (junior high school)	15	16.2	

Marital status	1 (unmarried)	13	40.5	0.095
	2 (married)	2	86.5	

**Table 4:** Comparison of the basic conditions of the two groups of patients.

Variable name	Variable meaning	Intervention group (*N* = 37)	Control group (*N* = 38)	*T*	*P*
Illness years	Course of illness	11.14 ± 7.88	9.63 ± 7.64	0.839	0.404
Complications	Number of complications	15.1 ± 1.54	1.16 ± 1.26	1.095	0.277

**Table 5:** Comparison of self-efficacy at the end of the two groups.

Variable name	Variable meaning	Intervention group (*N* = 37)	Control group (*N* = 38)	*T*	*P*
Self-efficacy	Initial self-efficacy	426 ± 0.72	4.04 ± 0.86	1.217	0.228
	Self-efficacy	4.45 ± 0.58	4.16 ± 0.66	2.032	0 046

**Table 6:** Specific comparison.

Variable	Intervention group	Control group	*T*	*P*
	(*N* = 37)	(*N* = 38)		
Healthy eating at the end of the term	0.79 ± 0.16	0.71 ± 0.17	1.372	0.174
Quality sleep at the end of the period	0.75 ± 0.17	0.69 ± 0.18	0. 482	0.631
Light exercise at the end of the period	0.70 ± 0.20	0.67 ± 0.23	0.262	0.794
High-intensity exercise at the end of the term	0.82 ± 0.18	0.81 ± 0.18	1.600	0.114
Follow the doctor at the end of the term	0.52 ± 0.27	0.43 ± 0.19	0.610	0.543
End-of-term blood glucose monitoring	0.88 ± 0.15	0.85 ± 0.24	2.302	0.021

**Table 7:** Comparison of HbA1c values at the end of the two groups.

Variable name	Variable meaning	Intervention group (*N* = 37)	Control group (*N* = 38)	*T*	*P*
HbAIc	HbA1c at the beginning of the period	7.23 ± 0.83	7.45 ± 0.97	−1.059	0.293
	HbA1c at the end of the period	6.79 ± 1.03	7.21 ± 1.19	−1.608	0.112

## Data Availability

No data were used to support this study.
